The article "Analysis and Prediction of Cross-Border e-Commerce Scale of China Based on the Machine Learning Model" was published in 2022. Journal: Comput Intell Neurosci.

# Analysis and Prediction of Cross-Border e-Commerce Scale of China Based on the Machine Learning Model

**DOI:** 10.1155/2022/7906135

**Published:** 2022-08-23

**Authors:** Qiaoping Chen

**Affiliations:** School of Foreign Studies, Yiwu Industrial and Commercial College, Yiwu, Zhejiang 322000, China

## Abstract

In the context of the rapid development of Internet technology, the integration of the world economy has been strengthened, and the continuous innovation of technology and foreign trade business forms has promoted the rapid development of cross-border e-commerce. Due to the lack of relevant data on cross-border logistics empirical research, this paper conducts a prediction study on the scale of China's cross-border e-commerce market based on machine learning models and combines the relevant financial reports of listed companies to determine the proportion of performance costs to turnover. Forecast of the scale of cross-border e-commerce in China. Combined with the total economic volume, industrial structure, domestic and foreign trade, online shopping development, people's life, and express development, the index system is established, and 11 indicators are initially established with reference to the selection principle of indicators. Combined with the research object, multiple regression and gray prediction methods are established. The relevant prediction model is tested, and the established model is tested to ensure the prediction accuracy. The forecast results show that by 2027, the size of China's cross-border e-commerce market will reach 30.8133 trillion yuan.

## 1. Introduction

Since the establishment of the Shanghai Free Trade Zone in 2013, China has established 11 free trade zones including Guangdong and Tianjin. In 2015, China proposed the Belt and Road development strategy. In the context of the national macro development strategy of the Belt and Road Initiative and the Pilot Free Trade Zone, China's cross-border e-commerce has become a dark horse in foreign trade. According to customs statistics, China's total import and export of goods in 2016 was 24.33 trillion yuan, a year-on-year decrease of 0.9 percentage points. While China's import and export trade declined, the scale of China's cross-border e-commerce transactions reached 6.3 trillion yuan in 2016, an increase of 23.5%. In the face of the rapid development of cross-border e-commerce, the State Council has also issued relevant guidelines to make an overall plan for the development of cross-border e-commerce, and the development of cross-border e-commerce in China has also entered a new stage of development.

Premier Li Keqiang emphasized a series of achievements in opening up in recent years and reviewed the progress of the Belt and Road Initiative. The inclusion of RMB into the SDR marks a new level of internationalization. Shenzhen-Hong Kong Stock Connect was launched import and export levels stabilized. The advanced experience of the Shanghai Free Trade Zone is also being comprehensively promoted in an orderly manner. Thanks to the promotion of policies, China's foreign trade development level has developed in a favorable direction as a whole. In the face of the complicated foreign trade situation, cross-border e-commerce, as a special form of foreign trade, has drawn much attention to its operation. Coupled with the active guidance and support of policies, the research on cross-border e-commerce is very valuable. Cross-border e-commerce logistics is an important part of cross-border e-commerce transactions, and the two depend on each other. At present, there are many obstacles and problems in cross-border logistics, which hinder the improvement of consumer experience and thus limit its development. Therefore, it is urgent to carry out research on cross-border logistics.

Foreign research on forecasting started earlier. In 1983, when Makridakis was studying problems related to time series, he conducted an empirical study on combined forecasting for the first time, and finally came to the conclusion that combined forecasting can effectively improve forecasting accuracy, and the more methods, the more accurate the forecast. The more accurate the prediction results [1]. In terms of the application of prediction methods, Terasvirta et al. [2] in 2004 used the monthly macroeconomic data of 7 countries for 47 months, using the smooth transition autoregressive model (STAR) and neural network (NN) model. In 2007 [2], Aburto and Weber [3] took the demand of supermarket commodities in Chile as the research object, using the ARIMA model and neural network. The model makes combined predictions, and the prediction results help supermarkets to effectively reduce the inventory level [3], and the practical application of prediction has achieved corresponding economic benefits. In 2017, facing the dynamic logistics demand, Sheu and Kundu [4] proposed a three-tier supply chain framework based on the Marr model. The logistics interaction model of the Kov chain and the validity of the established model were tested with the help of the logistics data of PetroChina, and the results proved the reliability of the model [4]. In terms of cross-border e-commerce, Gomez-Herrera et al. [5] in 2014 discussed the driving force and obstacle factors in the development of EU cross-border e-commerce. Studies have shown the convenience of cross-border e-commerce transactions, but also increase other related costs [5]. In 2015, Asosheh et al. [6] proposed a localization process for cross-border B2B e-commerce. The paper divides the process of cross-border B2B into three layers: message layer, business process layer, and content layer. Each level must have corresponding standard processes and corresponding solutions. Process optimization helps cross-border B2B e-commerce operate efficiently [6]. In terms of cross-border logistics, in 2013, Davis and Friske [7] took the United States and Canada as examples to study the impact of public-private partnerships on cross-border logistics using grounded theory. The quality of the operation of the environment logistics [7]. In 2014, Wong et al. [8] took the Pearl River Delta region of China as the research object and proposed the importance of bonded warehouses for cross-border logistics. On this basis, a PMS performance evaluation framework is proposed. The PMS framework includes four dimensions: time, cost, quality, and flexibility. Research shows that the PMS framework can help enterprises to improve competitiveness and resource allocation efficiency [8]. In 2016, Ai et al. [9] studied for the performance evaluation of cross-border logistics, a corresponding performance evaluation model is constructed using the two-sided market theory. On the other hand, it points out that cross-border payment is the bottleneck of cross-border e-commerce development and puts forward corresponding policy suggestions on cross-border payment [9].

The development speed of China's cross-border e-commerce is eye-catching, especially in academia. This field is a new research direction in recent years. Noticing the importance of cross-border logistics, more and more scholars are focusing on research-related issues of cross-border logistics [10–15]. The current research mostly focuses on the analysis of the status quo, solutions (overseas warehouses, bonded warehouses), and policy recommendations, and there is little empirical analysis [16, 17]. Therefore, the research purposes of this paper are two: one is to establish a corresponding market scale forecasting system, and with the help of the corresponding index system, to do a current research and short-term forecast on the scale of China's cross-border e-commerce market. The second is to make corresponding predictions on the scale of China's cross-border e-commerce logistics market. The theoretical significance of the research is to enrich the application scope of multiple regression forecasting and gray forecasting. Both prediction models are classic models, and when faced with new problems, the classic prediction models are adopted to enrich their applications. Another aspect of theoretical significance lies in enriching the empirical research on China's cross-border logistics. The empirical research based on data has reliable data sources, and the research conclusions are objective and have good guiding significance. The forecast of China's cross-border e-commerce market size and cross-border e-commerce logistics has important reference value for the government to formulate development plans for cross-border logistics and integrate logistics resources. With the deepening of China's opening to the outside world, the economic pillar effect of foreign trade has become more and more obvious. As a form of trade with the fastest growth in recent years, cross-border e-commerce has a good impact on the development of China's foreign trade guiding value.

## 2. Theoretical Background

### 2.1. Cross-Border e-Commerce

Cross-border e-commerce refers to a business form in which buyers and sellers in different countries use cross-border e-commerce platforms to reach purchase agreements, buyers pay for goods, and sellers are responsible for delivery and distribution. In a broad sense, it can be considered that foreign trade e-commerce means that buyers and sellers in different customs will digitize the traditional foreign trade process, complete the distribution with the help of international logistics, and finally achieve the purpose of the transaction. In a narrow sense, we can understand cross-border e-commerce as international retail. That is, the transaction activities of consumers in one country purchasing goods from other countries through cross-border e-commerce platforms. Cross-border e-commerce can be divided into cross-border export and cross-border import according to the logistics direction. In the cross-border export process, foreign goods are finally delivered to consumers or enterprises through e-commerce platforms, international payment companies, domestic and foreign customs, and domestic and foreign logistics companies. The cross-border import process is similar to the export process, but in the opposite direction. There is currently no mature theoretical system to support cross-border e-commerce, but the essence of cross-border e-commerce is international trade, and its economic essence lies in the international relationship between production factors circulation. The economic connotation of the development of cross-border e-commerce lies in reducing the mismatch between supply and demand markets, reducing the transaction costs of producers and consumers in the global market, and optimizing the allocation of resources.

### 2.2. Heckscher–Ohlin Model (H-O Model)

Heckscher–Ohlin (H-O) Model is the basic theory of international trade, it points out that resource difference is the fundamental reason for trade. In the process of international trade, a country should export its relatively rich products and import scarce products. The economic principle of the H-O model is shown in Figure 1. Suppose two countries realize commodity circulation through international trade, one country exports commodity *X* and imports *Y*, and the other country exports commodity *Y* and imports *X*. As the import and export proceed, the prices of the two commodities change accordingly, thus affecting the consumption. Equilibrium is achieved when the relative prices of the same commodity in the two countries are the same. The result of the equilibrium is that both sides of the trade increase the level of domestic consumption and gain benefits from international trade. For China, cross-border e-commerce, as a new form of international trade, can give full play to the advantages of China's resources and population and provide assistance for China's transformation and development.

### 2.3. Cross-Border Logistics

Cross-border logistics refers to logistics services carried out between different countries. From the definition of cross-border logistics, it can be seen that the two sides of the cross-border logistics trade cannot come from countries, and the goods traded need to go out of the country where the sender is located, and then complete the entry and exit procedures after arriving in the country where the consignee is located, and finally delivered to consumers through logistics and distribution. The entire process of cross-border logistics can be divided into three parts, domestic logistics in the country where the goods are sent, international logistics, and logistics and distribution in the country where the consumer is located. The difference between cross-border logistics and domestic logistics is that it needs to go through the domestic and destination country customs and will be subject to customs supervision. Therefore, the operation process is more complicated, and the operation requirements of enterprises are higher. At present, few enterprises can complete all cross-border logistics alone operate.

Compared with domestic logistics, the characteristics of cross-border logistics are as follows: (1) Cross-border logistics has a long timeliness. The most significant difference between cross-border logistics and domestic logistics is the geographical distance between the origin and the destination. In general, the transportation mileage of cross-border logistics is significantly longer than that of domestic logistics, which determines that the timeliness of logistics is difficult to guarantee. (2) The cost of cross-border logistics is high. Due to the increase in transportation mileage, the cost of logistics and transportation has increased significantly, eroding the profits of cross-border e-commerce, and thus increasing commodity prices and affecting consumer demand. (3) The cross-border logistics process is complex. Cross-border logistics involves cross-border trade, which involves a series of links such as domestic first-way delivery, customs clearance, and destination delivery. A flaw in one of these links will directly lead to the failure of the transaction.

## 3. Analysis and Prediction of Cross-Border e-Commerce Scale of China Based on Machine Learning Model

### 3.1. Establishment of a Forecasting Indicator System for the Scale of China's Cross-Border e-Commerce Market

For the scale of China's cross-border e-commerce market, we can use the corresponding statistical indicators to describe the scale of China's cross-border e-commerce transactions. The gross domestic product (GDP) is used to describe the economic aggregate index in the previous literature, and this index is also used in this paper. As far as industrial structure indicators are concerned, we usually use the added value of the tertiary industry or the ratio of the tertiary industry to represent the industrial structure of a specific region. For domestic and foreign trade, we use two indicators: total retail sales of consumer goods and total imports and exports. The Internet development indicators closely related to the development of China's cross-border e-commerce are described by the number of Internet users and the scale of online shopping users. We use the express volume and express business income to study the indicators of China's express delivery development. In addition, we use the per capita disposable income and consumption level of urban residents to describe the economic level of consumers. Therefore, we initially obtained the relevant indicators for the prediction of the scale of China's cross-border e-commerce market, as shown in Table 1.

### 3.2. Gray Relational Model

The gray correlation degree is a measurement tool to judge the degree of correlation between indicators. The principle is to judge the geometric similarity between the research sequence and the target sequence, so as to obtain the degree of association between the target systems. The precondition for calculating the gray correlation degree is to clearly describe the characteristic behavior variables and related factor variables of the research system and then determine the sequence of its corresponding variables according to the actual sample data. And build a matrix, and finally analyze the results according to the expertise in the target field.

The correlation coefficient refers to the degree of correlation between each target indicator and the reference indicator in each year, so there will be a value for each year. This results in too much information, which cannot well reflect the overall correlation between the influencing factor and the predictor at all times. Therefore, it is necessary to integrate the correlation coefficients of each year into a single value, so as to facilitate the comparison between the various factors. In this paper, the average value of each index over the years is selected to represent the degree of correlation, and the specific formula is:

(1) $$\begin{array}{c} R_{i}=\frac{1}{k}\sum_{i}^{n}p_{i}\left(k\right), \end{array}$$

where *R* is the degree of association, *k* is the number of indicators, and *p* is the impact value. Here, we take the average of the correlation coefficients of each indicator over the years as the final indicator correlation degree. As can be seen from Table 2, the priority order of strength and weakness affecting the scale of China's cross-border e-commerce is: express delivery business revenue *X*_11_, online shopping user scale *X*_7_, express delivery volume *X*_10_, total retail sales of consumer goods *X*_5_, tertiary industry added value *X*_4_, household consumption level *X*_9_, GDP *X*_1_, and per capita disposable income of urban residents *X*_8_. The correlation between these 8 factors and the scale of cross-border e-commerce in China is more than 0.65. It can be seen from Table 2 that these 8 factors have a high correlation with the market scale. In the following prediction model modeling of market size, in order to improve the prediction accuracy, according to the strong correlation principle of index selection, this paper selects 8 factors whose gray correlation degree is greater than 0.65 among the above 11 indicators as independent variables for modeling analyze.

### 3.3. Multiple Linear Regression Model for Predicting the Scale of China's Cross-Border e-Commerce Market

The first step in regression analysis is to identify independent and dependent variables. Usually, the object to be studied is the dependent variable, and the relevant factors are the independent variables. In this paper, the dependent variable is the size of China's cross-border e-commerce market, and the independent variables are the eight indicators selected in the previous section. Therefore, we construct a multiple regression model. Due to the multivariate brings computational difficulties. In order to solve this problem, this paper uses the data analysis software SPSS to complete the calculation. Let the random variable *Y* and the general variables *X*_1_, *X*_2_,…, *X*_*k*_ have the following linear relationship:

(2) $$\begin{array}{c} Y=\beta_{0}+\beta_{1}X_{1}+\beta_{2}X_{2}+\cdots +\beta_{k}X_{k}+\mu , \end{array}$$

where *β*_0_, *β*_1_, *β*_2_,…, *β*_*k*_ are the regression coefficients, *Y* is the explained variable, *X* is the explanatory variable, and *u* is the random error. Use the historical data and time *T* of each indicator to establish a univariate regression model, and finally obtain the forecast results from 2023 to 2027 with the help of formula (2). Combining with Table 3, it can be seen that by 2027, the size of China's cross-border e-commerce market will exceed 20 trillion mark, reaching 30.8133 trillion yuan. It shows that under the current macroeconomic situation and the slow recovery of the world economy, the scale of China's cross-border e-commerce market will achieve steady growth, and it also verifies that the forecast results are in line with objective facts.

## 4. The Impact of Intelligent Tourism Loop on Traffic between Scenic Spotsevelopment Environment of China's Cross-Border e-Commerce

### 4.1. Political Environment

With the development of e-commerce in China, the development of domestic e-commerce has entered a period of stable development. At this stage, the demographic dividend is no longer obvious. In order to pursue profit growth, domestic e-commerce companies will focus more on the shopping experience of consumers. In this process, the government's regulatory policy has played a crucial leading role from beginning to end. Therefore, in the process of studying cross-border e-commerce, we must pay attention to policy guidelines and policy orientations. The development of cross-border e-commerce is also inseparable from policy support to a certain extent.

As far as China is concerned, large-scale cross-border e-commerce emerged relatively late. Compared with domestic e-commerce, the development of cross-border e-commerce lags behind domestic e-commerce due to its special transaction model. However, in recent years, due to the attention of the capital market., the momentum of development is fierce, injecting new vitality into China's cross-border trade. In order to regulate the development of the industry, China has also issued corresponding policies and regulations in recent years. The promulgation of these policies and regulations not only points out the direction for the development of cross-border e-commerce, but also improves the legal environment, so that there are laws and rules to follow when dealing with relevant conflicts and disputes.

After interpreting the relevant policies, we found that the national macro level has a positive attitude toward the development of cross-border e-commerce in China and has created many convenient conditions. It can be seen that the development of cross-border e-commerce in China in recent years has attracted the attention of the state, and its impact on China's foreign trade has also been affirmed by the state. At the same time, the country has also seen discordant aspects in the development process and has issued relevant management rules and regulations. Under the guidance and supervision of policies, China's entry into the e-commerce market will inevitably make great strides in the direction of healthy development. After a transitional period, the new cross-border e-commerce policy will inevitably lead the industry to gradually become standardized. Under the guidance of policies and regulations, some backward small enterprises will inevitably be eliminated, corresponding market-leading enterprises will be cultivated, and industry innovation will be led to lead industry norms. In terms of delivery mode, bonded warehouses have natural logistics advantages, and centralized procurement of explosives is conducive to large-scale operations and lower operating costs, which is conducive to the healthy development of the cross-border e-commerce industry.

### 4.2. Economic Environment

The internationalization of the RMB aims to promote the international status of the RMB as a globally recognized currency for pricing, settlement, and reserves. In 2016, the RMB was officially included in the SDR. There are currently five currencies in the SDR currency basket, of which the US dollar accounts for the highest proportion, reaching 41.73%, followed by the euro, accounting for 30.93%, and the third is the RMB, accounting for 10.92%, the last Japanese yen (8.33%), and the British pound (8.09%).

The inclusion of RMB into the SDR is of strategic significance, and at the same time, it further accelerates the process of RMB marketization. The addition of the RMB to the SDR not only enhances the international currency status of the RMB, but also enhances the pricing power of the RMB in commodities. The impact of RMB internationalization on China's cross-border e-commerce is reflected in the payment and settlement links, and the corresponding currency advantages will gradually emerge. The internationalization of the RMB has provided very convenient basic conditions for the development of cross-border e-commerce in China.

Thanks to the continuous development of the global economy and the deepening of the degree of integration, cross-border e-commerce, as a brand-new trading method, benefits from the simplicity of its transaction links and reduces the operating costs of foreign trade price advantage. In particular, the Belt and Road national strategy has created a new situation for China's foreign trade. Taking this opportunity, China can allow more enterprises to go to the world through cross-border e-commerce and promote enterprises development to accelerate transformation and upgrading in the new foreign trade situation.

### 4.3. Social Environment

There are many reasons for the upgrading of people's consumption concept, one is the progress of society, the other is the rise of living standards, and the third is the improvement of the level of education for all. When domestic consumer goods cannot meet people's consumption needs, people naturally turn their attention to the world and look for satisfactory products around the world. Cross-border e-commerce provides convenient conditions for meeting people's needs, allowing people to understand commodity information around the world without leaving home, and meeting people's diversified consumption needs. The development of information technology and the change of consumption concepts have made Online shopping an extremely common thing and have been recognized by more and more consumers. Therefore, the upgrading of the consumption concept provides convenient conditions for the development of the industry.

The improvement of networking infrastructure and the popularization of mobile Internet have brought great network convenience to people. China's network infrastructure has developed from the earliest narrowband to the later low-speed broadband to the current high-speed optical fiber communication. China's Internet broadband level has developed by leaps and bounds, and the network scale and the scale of netizens are also expanding year by year. In terms of mobile Internet, with The big investment in 4G networks of the three major operators and the continuous expansion of the coverage of wifi hotspots in cities and operators have greatly improved the surfing environment of mobile terminals. The improvement of Internet infrastructure is an essential prerequisite for the entire e-commerce industry.

## 5. Conclusion

The research on China's cross-border e-commerce and cross-border logistics is still in its infancy, and the relevant research literature is still relatively small. This paper refers to the selection of indicators and method applications for regional logistics forecasting in the past, selects appropriate indicators to analyze China's cross-border e-commerce market, and indirectly predicts the market size of cross-border e-commerce logistics by predicting the scale of China's cross-border e-commerce market. The work done in this paper is as follows: (1) Indicator selection. In the process of index selection, we mainly refer to the relevant indicators of previous logistics forecasting and adjust them according to the characteristics of cross-border logistics. The corresponding indicators are initially selected from five aspects: total volume, industrial structure, online shopping development, people's life, and express delivery development. (2) Index test. Due to the strong subjectivity in the process of index selection, this paper selects gray correlation analysis to test the degree of correlation between each index and the size of the cross-border e-commerce market. Through the test, it is found that 8 indicators have passed the correlation analysis. In the forecasting process, we use these 8 indicators for analysis and forecasting. (3) Choose a forecasting method. There are also many commonly used market size forecasting methods. This paper refers to the previous research literature and combines its own academic ability to select multiple regression forecasting models and gray forecasting models for forecasting research. Based on the regression forecasting results and gray forecasting results, the final cross-border forecast is completed through comprehensive integrated forecasting. E-commerce market size forecast.

## Figures and Tables

**Figure 1:** Heckscher-ohlin model.

**Table 1:** Cross-border e-commerce market scale forecast indicator system.

The target layer	The primary indicators	The secondary indicators
China cross-border e-commerce market size forecast	Economic aggregate	Gross domestic product
	Industrial structure	The added value of the primary industry
		The added value of the secondary industry
		The added value of the tertiary industry
	Domestic and foreign trade	The total retail sales of social consumer goods
		Total import and export
	Online shopping development	Scale of online shopping users
	people's life	Per capita disposable income of urban residents
		Resident consumption level
	Express development	Express volume
		Express business income

**Table 2:** Gray correlation degree.

Index	*X *_1_	*X *_2_	*X *_3_	*X *_4_	*X *_5_	*X *_6_	*X *_7_	*X *_8_	*X *_9_	*X *_10_	*X *_11_
Correlation	0.6638	0.6455	0.6423	0.6904	0.6973	0.6126	0.8512	0.6521	0.6688	0.8014	0.9447

**Table 3:** Forecast result.

Time	2023	2024	2025	2026	2027
Value	20.61024	22.71897	25.22368	27.57899	30.81331

## Data Availability

The raw data supporting the conclusions of this study can be obtained from the corresponding author upon request.
